The article "Advance of Nano-Composite Electrospun Fibers in Periodontal Regeneration" was published in 2019. Journal: Front Chem.

# Advance of Nano-Composite Electrospun Fibers in Periodontal Regeneration

**DOI:** 10.3389/fchem.2019.00495

**Published:** 2019-07-10

**Authors:** Yu Zhuang, Kaili Lin, Hongbo Yu

**Affiliations:** ^1^Department of Oral and Cranio-Maxillofacial Surgery, Shanghai Ninth People's Hospital, College of Stomatology, Shanghai Jiao Tong University School of Medicine, Shanghai, China; ^2^Shanghai Key Laboratory of Stomatology, National Clinical Research Center for Oral Diseases, Shanghai Research Institute of Stomatology, Shanghai, China; ^3^Shanghai Key Laboratory of Stomatology, Shanghai Research Institute of Stomatology, Shanghai, China

**Keywords:** nano-composite, electrospun fibers, synthetic polymers, natural polymers, inorganic components, periodontal regeneration

## Abstract

Periodontitis is considered to be the main cause of tooth loss, which affects about 15% of the adult population around the world. Scaling and root-planning are the conventional treatments utilized to remove the contaminated tissue and bacteria, but eventually lead to the formation of a poor connection—long junctional epithelium. Therefore, regenerative therapies, such as guided tissue/bone regeneration (GTR/GBR) for periodontal regeneration have been attempted. GTR membranes, acting as scaffolds, create three-dimensional (3D) environment for the guiding of cell attachment, proliferation and differentiation, and play a significant role in periodontal regeneration. Nano-composite scaffolds based on electrospun nanofibers have gained great attention due to their ability to emulate natural extracellular matrix (ECM) that affects cell survival, attachment and reorganization. Promoted protein absorption, cellular reactions, activation of specific gene expression and intracellular signaling, and high surface area to volume ratio are also important properties of nanofibrous scaffolds. Moreover, several bioactive components, such as bioceramics and functional polymers can be easily blended into nanofibrous matrixes to regulate the physical-chemical-biological properties and regeneration abilities. Simultaneously, functional growth factors, proteins and drugs are also incorporated to regulate cellular reactions and even modify the local inflammatory microenvironment, which benefit periodontal regeneration and functional restoration. Herein, the progress of nano-composite electrospun fibers for periodontal regeneration is reviewed, including fabrication methods, compound types and processes, and surface modifications, etc. Significant proof-of-concept examples are utilized to illustrate the results of material characteristics, cellular interactions and periodontal regenerations. Finally, the existing limitations of nano-composite electrospun fibers and the development tendencies in future are also discussed.

## Introduction

Periodontitis causes the progressive destruction of periodontal tissues, and affects about 15% of the adult population worldwide. The periodontium is composed of gingiva (gum), alveolar bone, periodontal ligament (PDL), and cementum (Figure 1) (Bottino et al., 2012; Sowmya et al., 2013). Cementum and alveolar bone are mineralized tissues, and they mainly surround and support the teeth. Gingiva and PDL are fibrous tissues, and PDL, also called Sharpey fiber, anchors the cementum of tooth root to the adjacent alveolar bone (Melcher, 1976). Periodontal disease can lead to loss of teeth. The worldwide prevalence of this disease has led to great demand for effective therapies. The ultimate ideal outcome is to reconstruct the original hierarchical complex architecture of periodontium, including new cementum, alveolar bone and PDL, which is called periodontal regeneration (Bosshardt and Sculean, 2009; Ripamonti and Petit, 2009). Although defected periodontium can be restored partially in clinics now, complete periodontal tissue regeneration has not been successfully realized in humans, for reasons like oral hygiene, defect size, infection and many others (Polimeni et al., 2006). The weak innate regeneration ability of periodontal tissues demonstrates the demand for clinical therapies for periodontium regeneration.

**Figure 1:** Compositions of the periodontium. Adapted with permission from Chen et al. (2010a). Copyright 2010 Elsevier.

Conventional treatment, open flap debridement (OFD), provides more access for scaling and root-planning, which can remove the bacteria and contaminated tissue from root surface, while leading to the formation of a poor connection—long junctional epithelium. If left empty after OFD, epithelial cells and fibroblasts will firstly fill in the defects, which prevents the sequential regeneration of true periodontal tissues (Chen et al., 2010a). Therefore, regenerative therapies, such as guided tissue/bone regeneration (GTR/GBR) for periodontal regeneration, have been attempted.

GTR utilizes a barrier membrane to prevent epithelial cells and fibroblasts from migrating into defected space, and maintain sufficient space and time for the regeneration of alveolar bone, cementum and PDL (Zhang et al., 2007; Park et al., 2009). The non-degradable membranes utilized in clinics mainly include polytetrafluoroethylene (PTFE) membrane like Cytoplast® TXT-200 and titanium-strengthened PTEE membrane like Cytoplast® Ti-250, and the main shortcoming lies in its inability to degrade, requiring a second operation (Gentile et al., 2011). To avoid additional surgical procedures, attempts have been made to develop degradable membranes, and the majority of the membranes on the market are based on synthetic polymers like poly-caprolactone (PCL), poly lactic acid (PLA), polyglycolic acid (PGA), and their copolymers, etc. (Coonts et al., 1998; Donos et al., 2002; Hou et al., 2004), and natural polymer like collagen (e.g., from porcine skin, Bio-Gide®) (Bunyaratavej and Wang, 2001), mainly fabricated by melting or solvent casting approaches. However, there are inevitable disadvantages in current GTR membranes, like low attachment to the adjacent tissues, lack of antibacterial properties, and poor ability to enhance tissue regeneration (Behring et al., 2008). In addition, existing biodegradable membranes are weak in appropriate mechanical properties and controllable degradation rate (Jung et al., 2013).

GTR can be conducted in combination with bone grafts to prevent membrane collapse (Figure 2) (Chen et al., 2010a). Currently in clinics, bone grafts including autografts, demineralized freeze-dried allografts and bovine derived xenografts have been used to restore alveolar bone defects. However, pre-existing curative effects indicate that the commercial grafts can just fill in the periodontal bone defects, and perform poorly in promoting hierarchical structure regeneration because of poor osteoinductivity (Yang et al., 2009; Reynolds et al., 2010).

**Figure 2:** Schematic illustration of GTR membrane combined with bone grafts therapy for periodontal regeneration. Adapted with permission from Chen et al. (2010a). Copyright 2010 Elsevier. **(A)** Periodontal defect with loss of PDL and alveolar bone. **(B)** Bone grafts in the defected site. **(C)** GTR/GBR membrane covered on the grafts. **(D)** Sewing for closure of the wound.

The ideal membrane has yet to be developed for enhancing periodontal regeneration. GTR/GBR membranes, acting as scaffolds to emulate the ECM, might recruit stem cells and progenitors from the retaining healthy adjacent alveolar bone, PDL and blood, and promote the proliferation and differentiation of these stem cells into fibroblasts, osteoblasts, and cementoblasts (Larsson et al., 2016). They are required to stay in place for at least 4–6 weeks with appropriate mechanical, biocompatible and degradable properties to prevent soft tissue growing into alveolar bone defects (Veríssimo et al., 2010), and induce bone regeneration for optimized periodontal regeneration (Kikuchi et al., 2004).

To obtain membranes with optimal properties, like biocompatibility, biodegradability, osteoconductivity, even osteoinductivity and ability to promote cell attachment, proliferation and differentiation for periodontal regeneration, electrospinning technology utilizing synthetic or/and natural polymers has received increasing attention (Bottino et al., 2012; Liu et al., 2018). Biocompatible electrospun nanofibers have an innate advantage in mimicking natural ECM, controllable degradation rate and excellent mechanic properties by regulating relative parameters. The small pore size of electrospun membranes can effectively inhibit migration of fibroblasts across the membrane barrier. To meet multiple requirements for periodontal regeneration, different polymers and various additives like active bioceramics, growth factors, proteins, and drugs can be incorporated into electrospun nanofibers to obtain ideal properties.

To update the advantage of electrospinning technology for periodontal regeneration, different components of various synthetic and natural polymers as matrixes and inorganic components as bioactive additives for periodontal regeneration are reviewed in this paper. Functional growth factors, proteins for optimized osteogenesis activity, and drugs like antibiotics for better regulation of inflammatory microenvironment are described. The existing limitations of nano-composite electrospun fibers and the future development trends are also discussed.

## Electrospinning Technology for the Fabrication of Electrospun Fibers

Electrospinning has gained more and more attention for the reason that it is widely recognized as a powerful tool for fabricating nanoscale materials with controllable fiber diameter, porosity, ideal morphology, and optimized surface characteristics (Lu et al., 2018). Electrospinning utilizes a polymeric solution or melt to generate nanofibers in high electrostatic field. Various components can be added to obtain properties, and random/aligned nanofibers, core-shell structure can be obtained by modulating electrospinning setups (Figure 3) (Min et al., 2015; Wu et al., 2018). A typical electrospinning setup requires four components: a syringe pump (containing solution/melt/suspension to be electrospun), a spinneret with a metallic needle (as a capillary), a high-voltage power supply (for generation of high electrical voltage) and a grounded conducting collector (static plate or rotatable drum) (Min et al., 2015). A proper high voltage makes liquid droplet formed by the polymer solution electrically charged, and the droplet is stretched with electrostatic forces counteracting the solution surface tension. A “Taylor cone” can be formed at the key point of voltage, which is called the threshold voltage, and then a jet of liquid erupts from the surface (Jiang et al., 2015a). A jet of polymer charged fluid is pulled toward the grounded collection, with multiple nanofibers deposited and solidified, during which the solvent evaporates, leaving dry nanofibers on the collector (Dersch et al., 2003; Subbiah et al., 2005).

**Figure 3:** Schematic illustration for electrospinning process: **(A)** Various additives incorporated into polymer matrixes. **(B)** Uniaxial electrospinning setup. Adapted with permission from Min et al. (2015). Copyright 2015 Elsevier. **(C)** Coaxial electrospinning setup. Adapted with permission from Chen et al. (2010b). Copyright 2010 Elsevier. **(D)** Random nanofibers, **(E)** Aligned nanofibers. Adapted with permission from Qasim et al. (2017), doi.org/10.1016/j.dental.2016.10.003, by the terms of the Creative Commons Attribution License (CC BY), http://creativecommons.org/licenses/by/4.0. Copyright 2017 Elsevier. **(F)** Core-shell structure. Adapted with permission from Tang et al. (2016). Copyright 2016 Elsevier.

Moreover, to be applied in various fields, basic equipment can be improved, like using multiple needle syringes to obtain blended fibers, or rotatable mandrel collectors to fabricate hollow tube-like fibers. Generally, nanofibers made through electrospinning are unwoven if using a static collector, while electrospinning with two strips of electrodes or using a rotatable collector has the ability to fabricate aligned fibers (Li et al., 2003). Apart from uniaxial electrospinning, core-shell structure can be fabricated by coaxial electrospinning for drug loading and functionally graded membrane (FGM) with multi-functional layers that can be obtained by sequential electrospinning. To get the ideal physical-chemical-biological properties of fibrous scaffolds, proper polymer matrixes, suitable additives, optimized spinning processes (temperature, humidity, customized accessories, etc.), and appropriate post-processing should be taken into serious considerations during the electrospinning process.

Nanofibrous scaffolds possess unique properties, including high surface area to volume ratio, controllable porosity with interconnected pores, enhanced protein absorption, activation of specific gene expression and intracellular signaling, and promoted cellular reactions (Zafar et al., 2016). With larger surface to absorb proteins, nanoscale scaffolds present more binding sites to cell receptors (Stevens, 2005). Several bioactive components, such as bioceramics and functional polymers can be blended into matrixes to enhance regeneration ability, and functional growth factors, proteins and drugs can be incorporated to regulate cellular reactions and/or modify the local inflammatory microenvironment.

## Nano-Composite Electrospun Fibers in Periodontal Regeneration

Functional electrospun fibers can be obtained by blending various polymers together or incorporating functional components into the polymer matrixes. These composites are charming for reasons that these materials fabricated by electrospinning approach display good mechanical, bioactive and biological properties compared with the pure polymer matrixes. Various types of nano-components are summarized in Table 1.

**Table 1:** Various types of nano-composite electrospun fibers.

**Types of additives**	**Bioactive additives**		**Polymer matrixes**	**Advantages**	**Directions for future development**	**References**
Ceramics	Ca-P based components	HAp nanoparticles	PCL; COL; CS; SF; cellulose; PLA; GEL; PLGA	Major constituent of natural bone; promoting osteogenesis	Finding proper proportion to improve mechanical properties	Bottino et al., 2011; Wu et al., 2014; Lai et al., 2015; Tang et al., 2016; Ao et al., 2017
		β-TCP	PGS; PCL; CS	Ideal resorbability; promoting osteogenesis	Improving diameter, porosity, and contact angle	Masoudi et al., 2017
	Ca-Si based components	BGs	PCL; CS; GEL; COL; PVA	Releasing Ca^2+^ ions and silicate; promoting osteogenesis	Enhancing efficacy of osteogenesis activity	Zhou et al., 2017b
	Oxides	ZnO	PCL	Antibacterial activity; promoting osteogenesis	Ensuring non-toxicity	Nasajpour et al., 2018
		CaO	PCL	Promoting osteogenesis	Improving mechanical properties	Münchow et al., 2015b
Carbon-based components		MWNTs	PLGA; PLA	Improving the strength and toughness; promoting osteogenesis	Solving non-resorbability	Zhang et al., 2018
		GO	P34HB	Improving mechanical strength; antibacterial activity; promoting osteogenesis	Solving non-resorbability	Zhou et al., 2017a
Metal components		AgNPs	CS	Excellent antibacterial activity	Ensuring non-toxicity	Shao et al., 2017
		AuNPs	/	Promoting osteogenesis	Further exploring AuNPs incorporated nanofibers	Jadhav et al., 2018
Drugs	Antibiotics	MNZ; ampicillin; amoxicillin; tetracycline hydrochloride; doxycycline hydrochloride; tinidazole	PLA; PLGA; GEL; COL	Ideal antibacterial activity	Improving releasing profile	Reise et al., 2012
	NSAIDs	Ibuprofen; piroxicam	PCL; CS; PVA	Anti-inflammation activity	Improving releasing profile	Batool et al., 2018
Growth factors		BMP; PDGF	COL	Promoting osteogenesis	Enhancing delivery efficacy and biological activity	Ho et al., 2017
Proteins		AMPs;	PLGA; CS; GEL	Antibacterial activity	Guaranteeing biological activity	He et al., 2018b
		Fibronectin	PLGA	Enhancing cell recognition	Improving connection method	Campos et al., 2014

### Nano-Composite Electrospun Fibers Blended With Polymer Matrixes

Synthetic polymers have good mechanical properties and electrospinnability, but poor biological characteristics. It is a promising way to blend natural polymers with inherently good bioactive properties with synthetic polymers to promote cellular reactions in periodontal regeneration.

Polysaccharides, like chitosan, cellulose and alginate, etc., are attractive polymers in tissue engineering applications for their ideal biological properties and easy accessibility. Chitosan (CS) is a natural polymer, degraded into glycosylated collagen and chondroitin sulfate *in vivo*, which is widely studied for periodontal regeneration due to its excellent biological performance or, in other words, biocompatibility, biodegradability, and inherent antimicrobial properties (Eugene and Lee Yong, 2003; Lee et al., 2009). It was reported to improve osteogenic differentiation by means of enhancing mitogenic property of osteoblastic cells for bone regeneration (Peter et al., 2010; Anitha et al., 2014). Amine groups of chitosan offer a positive-charged surface, and chitosan is a relative hydrophilic material, thus, being able to promote protein adsorption and cell adhesion. But it lacks mechanical stability and solubility in water, and leads to the brittle nature of scaffolds. It can be blended with different synthetic polymers, like PLA (Shen et al., 2018), PCL (Masoudi et al., 2017), and bioceramics, etc. to make up for these shortcomings.

Cellulose, with good biocompatibility and biodegradability, is easily obtained from the natural world. Electrospun bacterial cellulose (BC)/hydroxyapatite (HA) nanofibers were prepared to promote osteogenic differentiation of stem cells (Ao et al., 2017). With ideal mechanical properties like high tensile strength and elastic modulus, BC is a promising material in GTR (Zhang et al., 2018). Alginate, similar in structure to glycosaminoglycan (GAG), the component of ECM, is one of most useful natural polymers in the biomedical field. Previous studies indicated that the addition of alginate could promote cell viability and osteogenic differentiation of stem cells (Hu and Yu, 2013;Ataie et al., 2019).

Structure proteins are vital components in ECM, and they are capable of enhancing the mechanical and biological properties of nanofibers, which make them promising GBR materials. Collagen (COL) shows good biological properties like high biocompatibility, good bio-affinity and resorbability, which can make up for the drawback of polyester in poor cell response, but it is insufficient in mechanical properties and dimensional stability (Liao et al., 2005). It degrades rapidly, and cannot shield the defected space efficiently because of its quick collapse (Bottino et al., 2011). Membranes based on collagen need to be further crosslinked, or blended with other polymers and additives like nHA (Wu et al., 2014) and bioactive glass (Zhou et al., 2017b) to overcome these drawbacks. Collagen was also electrospun on a chitosan basement to fabricate a bi-layered collagen/chitosan membrane for periodontal GBR (Lotfi et al., 2015).

In addition to collagen, there are many other proteins. Tussah silk fibroin (TSF), abundant in Arg-Gly-Asp motif and Asp, Ala, can be used to enhance cell adhesion. The addition of TSF can also improve mechanical properties like tensile strength (Shao et al., 2016). Zein, a native protein extracted from corn, has good biocompatibility and electrospinnability. However, the hydrophobicity of zein results in low cell affinity. It can be blended with the hydrophilic polymers, like gelatin, to overcome this disadvantage (Yang et al., 2017). He et al. (2017) constructed core-shell nanofibers utilizing zein as shell structure for its high hydrophobicity. Metronidazole was embedded in the core structure, and the hydrophobic polymer was used to prolong drug release.

Gelatin (GEL) has a structure similar to natural collagen, and possesses bio-signal groups which can enhance proliferation of various cells (Behring et al., 2008). It has been widely explored in tissue regeneration for its ideal biocompatibility and low immunogenicity. However, the high hydrophilicity of gelatin brings dissolubility in organic solution, thus it is attempted to be blended with various synthetic polymer like PCL (Xue et al., 2015; Kim et al., 2016; Ke et al., 2017), PLA (Bottino et al., 2011) and other natural polymers like zein (Yang et al., 2017) for enhanced solubility in spinning solvents and better electrospinnability.

For better electrospinnability and mechanical properties, synthetic polymers are widely utilized in electrospun GBR membranes. PCL is a biocompatible polyester with extraordinary mechanical properties, non-toxicity and ease of being electrospun into nanofibers (Shor et al., 2007). Despite the advantages described above, there are still some drawbacks. PCL increases hydrophobicity when the fiber diameter is electrospun into nanoscale, therefore it lacks in cell-recognizing sites, and leads to slower degradation rate and a lower expression of alkaline phosphatase (ALP) (Calvert et al., 2005). Chitosan blended with PCL provides a feasible strategy to overcome these disadvantages. The addition of hydrophilic chitosan into PCL matrix can lower its hydrophobic behavior and improve cell attachment. Furthermore, good miscibility doesn't constitute a requirement of any toxic crosslinking agents to crosslink them, unlike blends between PCL-gelatin and PCL-collagen (Shalumon et al., 2013; Nivedhitha et al., 2016; Masoudi et al., 2017).

PLA, as a biocompatible polyester, has been widely utilized in periodontitis treatment. Previous studies indicate that PLA can cause tissue inflammatory reaction due to its acidic degradation products. Negative effects can be exerted on the periodontal regeneration by acidic environment, and a relatively low pH value can lead to gingival inflammation (Bickel and Cimasoni, 1985; Patel et al., 2016). In addition, PLA is poor in hydrophilic property (Li et al., 2006). To overcome these disadvantages, Shen et al. (2018) embedded chitosan, the natural alkaline polymer, with PLA by electrospinning approach to improve its hydrophilicity and reduce acid products.

Co-polymers can take full advantages of both polymers, and they are extensively studied to explore materials with better properties. To improve the degradation rate of PLA, glycolic acid, which has analogous structure and faster degradation rate, can be incorporated into PLA chains to construct poly (lactide-co-glycolic acid) (PLGA), and to match repairing period of alveolar bone after periodontal regeneration therapy (6–12 months) (Park et al., 2009; Zhou et al., 2012). PLGA has the ability to regulate the degradation rate and improve the mechanical properties of PLA for bone regeneration (Lyu et al., 2013). However, PLGA has some disadvantages including weak hydrophilicity, cell adhesion, and acidic degradation products. Functional proteins (Campos et al., 2014), cellulose and multiwall carbon nanotubes (MWNTs) (Zhang et al., 2018) were added into PLGA nanofibers to improve cellular affinity, bioactivity, osteoconductivity and reduce aseptic inflammation. Additionally, it was reported that the incorporation of soluble eggshell membrane protein (SEP) could improve the electrospinnability and mechanical strength of PLGA (Jia et al., 2012). Poly (glycolic acid) (PGA) has good biocompatibility, but fast degradation rate by hydrolysis effect. While poly (butylene succinate) (PBS) degrades slower if compared with PGA, it has poor biological properties. Thus, the novel material poly (butylene succinate-co-glycolate) (PBSGL), based on PBS and PGA, was synthesized by Pajoumshariati et al. to take use to their advantage and make up for drawbacks (Pajoumshariati et al., 2018). Electrospun PBSGL membranes, with tunable hydrolytic rate, were proved to possess better mechanical and biological properties (Pajoumshariati et al., 2018).

In previous studies, multiple synthetic polymers have been utilized in electrospinning process for GBR application. Polyethylene oxide (PEO) could enhance viscosities of polymer solutions (Qasim et al., 2017), and was woven into nanofibers with proper morphologies (Hu and Yu, 2013). He et al. constructed naringin loaded polyvinylpyrrolidone (PVP) as a core fiber, which possessed good biocompatibility (He et al., 2018a). Poly (vinyl alcohol) (PVA) has good biodegradability and non-toxicity, and its films are uniform, thick, and foldable, which makes it effective in drug delivery system. Farooq et al. (2015) fabricated novel electrospun chitosan/HA/PVA membrane to load drug for GBR application.

Various synthetic and/or natural polymers can be blended and electrospun into nanofibers. Apart from different components affecting biological properties of nanofibers, alignment, topological, and mechanical cues might also have influence on the outcomes of alveolar bone and PDL regeneration. To achieve aligned PDL regeneration, the effect of the alignment form of nanofibers on cell bio-reactions has received increasing attention (Jose et al., 2009).

Jiang et al. (2015b) incorporated oriented biodegradable poly (caprolactone)-poly (ethylene glycol) (PCE) electrospun nanofibers mats into porous chitosan to realize the aligned PDL regeneration. The scaffolds were tailored into cross-sectioned slices, put against the exposed root surfaces, and then bovine-derived porous xenograft Bio-Oss was implanted to fill in the alveolar bone defect to immobilize the scaffolds. The rat periodontal defects regenerated PDL-like tissue arrangement after 2 months, and showed that aligned groups had more concentrated angles whose characters were closer to native PDL. Higher collagen I/collagen III ratio and more fibrous tissue formation were observed against random groups. These studies indicated that aligned nanofibers embedded scaffolds could enhance infiltration, viability, and expression of periostin of rat bone marrow mesenchymal stem cells (BMSCs), and led to more organized arrangement of regenerated PDL (Figure 4).

**Figure 4:** Process of aligned nanofibers embedded scaffold for organized PDL regeneration. Adapted with permission from Jiang et al. (2015b). Copyright 2015 Elsevier.

It is well-known that topological and mechanical cues play critical roles in the cell line of differentiation of periodontal ligament cells (PDLCs). PDLCs are exposed to mechanical pressure caused by occlusal forces. To study the effects of simultaneous topological and mechanical cues on the cell alignment and protein expressions of PDLCs, Kim et al. (2016) cultured PDLCs on aligned and random PCL/gelatin scaffolds, respectively under mechanical-stressed condition. The results showed that the cyclic uniaxial stretch and nanofiber alignment brought effects on differentiation orientation of PDLCs and led to higher expression of periostin, tenascin-C and TGF-β1 in aligned groups, which indicated the enhanced potential of PDLCs for ligamentogenesis with aligned fibers. But no unified conclusion on the effect of cyclic uniaxial stretch and nanofiber alignment on the reaction of PDLCs was reached, which needs to be further studied.

Random nanofibers are usually applied in alveolar regeneration, while aligned nanofibers perform better in organized PDL regeneration. To realize the simultaneous regeneration of both alveolar bone and aligned PDL, Qasim et al. (2017) fabricated a tri-layered membrane (Figure 5) consisting of random and aligned PEO-doped chitosan nanofibers, respectively. The aligned layer was designed for ligament and the random layer for alveolar bone. The histological results showed a large proportion of cell infiltration but a disorganized matrix deposition in random fibers group, while more organized deposited matrixes were observed in aligned fibers group. Therefore, a tri-layered membrane with different layer characteristics shows a possible way for simultaneous alveolar bone and aligned PDL regeneration.

**Figure 5:** Schematic diagram of a tri-layered membrane for simultaneous alveolar bone and aligned PDL regeneration. Adapted with permission from Qasim et al. (2017), doi.org/10.1016/j.dental.2016.10.003, by the terms of the Creative Commons Attribution License (CC BY), http://creativecommons.org/licenses/by/4.0. Copyright 2017 Elsevier.

### Nano-Composite Electrospun Fibers Blended With Inorganic Components

#### Nano-Composite Electrospun Fibers Blended With Ceramic Components

The strategy of polymer combined with bioceramic components was inspired by the nature hybrid structure of bone matrix: a complex composite constructed by organic collagen fibers and hydroxyapatite (HAp). Bioceramics, such as HAp nanoparticles and bioactive glasses (BG) can be incorporated into the electrospun fiber matrixes to promote bioactivity and biological-physical-chemical properties, such as osteoconductivity, osteoinductivity, and to emulate the native inorganic bone components (Heinemann et al., 2010; Yeo et al., 2011; Qasim et al., 2015). For better alveolar bone regeneration in periodontium restoration, bioceramics can be incorporated into natural and/or synthetic polymeric scaffolds, and the composite scaffolds show enhanced osteoconductivity in comparison with the single-component polymeric scaffolds.

##### Blended with Ca-P based components

*Hydroxyapatite (HAp) nanoparticle component*. HAp, with molecular formula Ca_10_(PO4)_6_(OH)_2_, is considered as the most thermodynamically steady synthetic calcium phosphate ceramic. It is biocompatible, bioactive and osteoconductive (Yang et al., 2009). It is the major constituent of natural bone, and has been widely applied in the bone repairing field. However, it is impossible to use HAp alone as scaffold material due to its brittleness. A large amount of researches have proved that HAp incorporated into electrospun nanofibers can improve their mechanical properties, proliferation and mineralization of osteoblasts (Prabhakaran et al., 2009; Zhang et al., 2017).

The incorporation of HAp can effectively promote bone regeneration. Compared with COL/PCL electrospun nanofibers, the incorporation of HAp nanoparticles could promote the expression of bone-related markers of PDLCs, such as alkaline phosphatase (ALP) and osteocalcin (OCN), and it showed possible applications in GBR in periodontium restoration (Wu et al., 2014). The stimulation of nHA on the proliferation, differentiation and mineralization of human mesenchymal stem cells (hMSCs) was also observed in CS/silk fibroin (SF) based electrospun fiber membranes, and the nano-composite electrospun fibers with 30 wt.% nHA were ideal for GBR (Lai et al., 2015). Ao et al. (2017) added activated native cotton cellulose into the well-dispersed nHA suspensions and obtained aligned nanofibers utilizing the high-speed rotating collector. The result showed that the addition of nHA could remarkably enhance the mechanical property of the membrane, and promote cell proliferation. Incorporation of nHA might not lead to cell cytotoxicity or affect nanofiber alignment adversely.

The functionally graded membrane (FGM) was explored for tailoring different layer properties to fabricate a material system with ideal physical, chemical and mechanical properties to optimize periodontal regeneration (Chen et al., 2013). Bottino et al. (2011) carried out a sequential multilayer electrospinning process to design a FGM composed of a core layer and two surface layers, respectively interfaced with bone and epithelial tissues for GBR, which showed to be promising in solving the shortcomings of currently available membranes, like weak mechanical property and poor osteoinductivity. In this multilayer membrane, the core layer was composed of a poly(DL-lactide-co-ε-caprolactone) (PLCL) layer surrounded by two ternary PLCL/PLA/GEL blended layers to provide ideal mechanical properties. The surface layer designed to be interfaced with bone consisted of PLA/GEL and nHAp to mimic natural collagen-HAp bone matrix to promote bone regeneration, while the layer designed to be interfaced with epithelial tissues had the PLA/GEL as matrix, loaded with metronidazole (MNZ) to combat periodontal pathogens (Figure 6).

**Figure 6:** Schematic diagram of the FGM for periodontal regeneration. **(A)** Membrane used for GBR. **(B)** The core layer (CL) and the functional surface layers (SLs), respectively interfaced with bone (n-HAp) and epithelial tissues (MNZ). Adapted with permission from Bottino et al. (2011). Copyright 2011 Elsevier.

Ideal GTR membranes require various properties, like barrier ability, bone regeneration activity, and inflammatory microenvironment regulation, etc. To meet these requirements, different additives need to be incorporated into the nanofibers, but for a more effective release and function of these additives, they should not be blended simultaneously in one single spinning solution. Coaxial electrospinning technology is a promising strategy to fabricate core-shell structure, making it possible to load different additives in core and shell, respectively for different purposes for regeneration. Tang et al. (2016) fabricated PLGA/HA (core)-collagen/amoxicillin (shell) membrane by coaxial electrospinning for GTR. The core consisting of PLGA/HA was designed to prevent fibroblasts growing into defected space, and enhance bone regeneration, and at the same time the shell composed of collagen/amoxicillin was aimed to enhance wound healing process.

*Beta tri-calcium phosphate (β-TCP) component*. Beta tri-calcium phosphate (β-TCP) has been widely applied in bone repair and GBR membranes for its excellent osteoconductivity and ideal resorbability, which are vital properties for required bone regeneration (Yang et al., 2015). It can be blended into various polymer matrixes to promote physical and mechanical properties along with cell reactions. Masoudi et al. (2017) fabricated a two-layered membrane by electrospinning method in which one layer used poly (glycerol sebacate) (PGS)/PCL and β-TCP for GBR and another one containing PCL/PGS and chitosan functioned for GTR. In particular PGS, as an elastomeric polymer, can provide flexibility for the GTR/GBR membrane (Zaky et al., 2014). The results suggested that the membrane containing 10 wt.% β-TCP showed an overall better performance in contact angle, hydrophilicity, mechanical properties, proliferation and ALP activity of human fetal osteoblasts (hFOBs). Furthermore, incorporation of chitosan into PCL/PGS nanofibers could promote GTR barrier properties, including the reduction of fiber diameter, porosity and contact angle.

##### Blended with Ca-Si based components

Bioactive glasses (BGs) are a typical group of Ca-Si based inorganic materials containing SiO_2_-CaO-P_2_O_5_ networks. The Ca-Si based materials with special components possess excellent osteoconductivity and even osteoinductivity (Murakami et al., 2017). BGs have been developed into various kinds of glasses and glass-ceramics. They perform well in small bone defect repair and are able to provide appropriate environment for the cultured cells to grow naturally like HAp. Its dissolution products have the ability to enhance the cell proliferation and activate the gene expression of osteoblasts (Xia et al., 2007). Therefore, BGs have been widely selected as bioactive components to be blended into various biodegradable electrospun polymers for bone tissue engineering applications, such as PCL/chitosan (Shalumon et al., 2013), PCL/gelatin (El-Fiqi et al., 2015) and PVA (Shankhwar et al., 2016), etc.

A biomimetic fish Col/BG/CS nano-composite electrospun nanofiber membrane was developed by Zhou et al. (2017b). The results revealed that the incorporation of BG promoted cell viability and gene expression of RUNX-2, ALP, OPN and OCN of PDLCs. Moreover, the *in vivo* results using the periodontal defect model in beagle dogs showed that much more new bone formed and less inflammation presented in the Col/BG/CS membrane group when compared with the Col/CS control group.

Compared with the traditional BG, the mesoporous bioactive glass nanoparticles (mBGn) possessed excellent ability for bone tissue regeneration due to prominent bone regeneration activity. The release of Ca and Si ions from mBGn could enhance the differentiation of stem cells or progenitors into osteoblasts (El-Fiqi et al., 2013). El-Fiqi et al. (2015) incorporated mBGn loaded with osteogenic drug Dexamethasone (DEX) into PCL/gelatin matrix by electrospinning method. Compared to the pure biopolymer matrix, the addition of mBGn enhanced the mechanical tensile strength, elasticity, and hydrophilicity. Moreover, the sustainable release of DEX further accelerated the proliferation and osteogenic differentiation of PDLCs.

HA and BG are both widely used for bone regeneration, but great attention has been devoted to determining which one performs better. Shalumon et al. (2013) compared the electrospun composite nanofiber membranes of nHA/PCL/CS (PCH) and nBG/PCL/CS (PCB) with the same amount (3 wt.%) of nHA and nBG. The results showed that both nHA and nBG could apparently enhance the ALP activity of human periodontal ligament fibroblast cells (hPDLFs), while the incorporation of nBG showed superior performance in the adhesion and proliferation of hPDLFs and osteoblast like cells (MG-63 cell lines). A similar phenomenon was also observed by Sunandhakumari et al. (2018). These studies indicate that, compared to nHA, mBG performs better in enhancing viability, attachment, proliferation and differentiation of osteogenic-relative cells.

##### Blended with oxide components

Periodontitis is an infective disease, in which bacteria release toxins, and the periodontium is then destructed. The main treatment strategy in clinics is topical antibiotics therapy, but the undesirable effects of antibiotics severely inhibit the curative effects. Therefore, it is important to control the release of antibiotics to regulate the inflammatory environment in periodontal regeneration. Incorporating antibacterial materials into electrospun nanofibers is a promising way due to controllable antibacterial function and enhanced bone regeneration activity at the same time. ZnO particles have potentials to introduce antibacterial activity and improve the osteoconductivity (Augustine et al., 2014; Münchow et al., 2015a). Nasajpour et al. (2018) incorporated ZnO into PCL by electrospinning method with ZnO concentrations of 0, 0.5, and 1 wt.%, respectively. *In vitro* periodontal ligament stem cells (PDLSCs) culture results indicated that PCL blended with 0.5 wt.% ZnO showed the optimal properties of cell viability, mineralization ability, and bone-related gene expression of Runx2, OCN, and ALP. Furthermore, *in vitro Porphyromonas gingivalis* culture proved that ZnO incorporated PCL membrane possessed excellent antibacterial activity. In conclusion, this novel membrane not only has antibacterial activity, but also has the ability to improve the osteoconductivity, which can makes it a promising candidate to regulate inflammatory environment and promote bone regeneration in periodontal regeneration.

Münchow et al. (2015b) incorporated CaO into PCL by electrospinning with different concentrations of CaO at 0, 5, 10, and 15 wt.%, respectively. The mechanical properties reduced progressively with the increase of CaO concentrations. The CaO-loaded membranes did not provide consistent antibacterial activity, while they increased the viability and osteogenic differentiation of MC3T3-E1. It is important to decide the appropriate type and concentration of oxide added into nanofibers during the electrospinning process to guarantee the biocompatibility of the implanted material.

#### Nano-Composite Electrospun Fibers Blended With Carbon-Based Components

Multiwall carbon nanotubes (MWNTs) have received great attention for their excellent mechanical properties, biocompatibility and stability for tissue engineering. Zhang et al. (2018) used bacterial cellulose (BC) membrane as lower membrane to collect electrospun PLGA/MWNT nanofibers to fabricate a bi-layered composite membrane, constructed by long, continuous fibers and weaved into a 3D network structure. The addition of MWNT remarkably improved the strength and toughness of the PLGA nanofiber scaffolds. Histological results of periodontal defect model tests showed that in PLGA/MWNT/BC composite membrane group, more newly formed PDL was found adjacent to new alveolar bone, and more collagen fiber bundles imbedded in the cementum and much more newly formed alveolar bone could be observed than in control group, indicating a greater ability to promote periodontal regeneration using MWNTs as additives.

It is also a strategy to blend MWNTs with HA to bring higher bioactivity. Mei et al. (2007) designed a PLA/MWNTs/HA composite GTR membrane in which the MWNTs and HA nanoparticles uniformly dispersed among the membrane. Comparing with the single PLA group, the addition of MWNTs and HA improved degradation property, and accelerated the adhesion and proliferation of PDLCs, at the same time the ingrowth of gingival epithelial cells was inhibited.

Graphene oxide (GO), derived from graphene, has received great attention in bone regeneration for its prominent mechanical strength, antibacterial property and capability of promoting osteogenic differentiation (Luo et al., 2015). Zhou et al. (2017a) fabricated electrospun P34HB/GO nanofibers, and the results indicated that GO could enhance tensile strength and Young's modulus of the membrane, and promote bone regeneration *in vivo*.

#### Nano-Composite Electrospun Fibers Blended With Metal Components

Various metal nanoparticles with different characteristics can be incorporated into nanofibers to improve membrane properties like antibacterial activity and bone regeneration activity, etc. Silver nanoparticles (AgNPs), which possess excellent antibacterial properties, show 1.4- to 1.9-times stronger antibacterial properties compared with silver ions (Ingle et al., 2008). Moreover, AgNPs have a much lower tendency to induce bacterial resistance compared with classical antibiotics (Sondi and Salopeksondi, 2004). Shao et al. (2017) fabricated a chitosan-based membrane blended with AgNPs. The results of antibacterial property evaluation revealed that AgNPs could have sustained antibacterial properties against *Porphyromonas gingivalis* and *Fusobacterium nucleatum* in a dose-dependent manner. Furthermore, appropriate amounts of AgNPs added into chitosan-based membranes did not cause noticeable cytotoxic effects on PDLCs, and the incorporation of AgNPs did not exert adverse influences on soft tissue responses. However, the safety intake amount of the AgNPs should be taken into consideration seriously.

Gold nanoparticles (AuNPs) were proved to have the potential to promote the differentiation of hPDLSCs into osteoblasts, increase their osteogenic-related expression of ALP, OCN, COL1, and RUNX2 via MAPK signaling pathway (Niu et al., 2017; Jadhav et al., 2018), while AuNPs incorporated electrospun fiber scaffolds still require more exploration in bone regeneration.

### Nano-Composite Electrospun Fibers Blended With Drugs, Growth Factors and Proteins

In the treatment for periodontitis, it is a feasible approach to incorporate multiple drugs into nanofibers to realize periodontal regeneration and anti-inflammation simultaneously. Anti-inflammatory agents can activate signaling cascades and trigger the healing process. Additionally, drugs loaded electrospun nanofibers can bring in remarkable characteristics, such as high loading capacity, high surface area to volume ratio and easy modulation of drug release profile.

Antibiotics, among the most useful drugs in clinics, are increasingly utilized in periodontal regeneration. Clinicians view metronidazole (MNZ) as the gold standard for the treatment of anaerobic infection, which is the main infection form of periodontitis. Reise et al. (2012) fabricated MNZ loaded electrospun PLA membrane, and found that this membrane could significantly inhibit the viability of periodontopathogenic species *F. nucleatum* and *P. gingivalis* for up to 2 days. Sequential electrospinning to fabricate FGM (Bottino et al., 2011) and coaxial electrospinning to construct core-shell structure (Tang et al., 2016) were utilized to incorporate MNZ into nanofibers for better drug delivery. Additionally, multiple drugs were added into nanofibers in attempts to assist periodontal regeneration, including ampicillin (Schkarpetkin et al., 2016), amoxicillin (Furtos et al., 2017), tetracycline hydrochloride (Ranjbar-Mohammadi et al., 2016), doxycycline hydrochloride (Debridement, 2016), and tinidazole (Khan et al., 2017), etc.

One of the purposes of periodontal treatment is to inhibit inflammatory reaction. Sustained release of prostaglandin (PG) during periodontal wound healing process exerts adverse effects on periodontal regeneration. Non-steroidal anti-inflammatory drugs (NSAIDs), like ibuprofen (Batool et al., 2018) and piroxicam (Farooq et al., 2015), can inhibit the activity of cyclooxygenase (COX), thus blocking arachidonic acid (AA) being converted into PG.

Growth factors can be used to promote osteogenesis of alveolar bone. Bone morphogenetic proteins (BMPs) were widely reported to enhance bone reconstruction in GBR (Shalumon and Jyh-Ping, 2015). Ho et al. (2017) incorporated platelet-derived growth factor (PDGF), a potent mitogen, into the nanofibers to facilitate alveolar ridge regeneration.

Functional proteins are also promising candidates to improve anti-bacterial and biological properties of materials. Antimicrobial peptides (AMPs) have a broad spectrum of antibacterial activity, distinguished from conventional antibiotics, which may result in bacterial resistance. He et al. (2018b) incorporated AMP-loaded PLGA microspheres into electrospun chitosan/gelatin nanofibers, which maintained the continuing release of Pac-525 to promote anti-bacterial activity. Fibronectin (FN) is a ligand–integrin affinity protein that can be found in ECM and cell membranes. It can aggregate adjacent cells by Arg-Gly-Asp (RGD) motif, and create binding sites to promote cell recognition. Campos et al. (2014) deposited FN onto hydrolyzed PLGA nanofibers to promote the bioactivity of scaffolds.

## Conclusions and Further Perspectives

Periodontitis is a chronic infection disease, which requires effective treatments for clinical applications. Conventional OFD can result in only weak epithelium connection, without affecting native periodontium structure. GTR is a promising method to promote the complex reconstruction of periodontium. Existing commercial GTR membranes still have no desirable curative effects, and have innate disadvantages, like poor mechanical property, inappropriate degradation rate and weak ability in promoting hierarchical periodontium regeneration, etc. Novel GTR membranes are required to possess three main properties to meet clinic requirements:

1. Proper degradability, mechanical properties and biocompatibility;
2. Optimized alveolar bone and organized PDL regeneration activity;
3. Antibacterial activity.

Electrospinning technology is prominently efficient in the fabrication of GTR membranes. Different polymers and various additives, soluble in relative solvents, can be subsequently electrospun into composite nanofibers. Electrospun nanofibers possess innate advantages in promoting periodontal regeneration, including high surface area to volume ratio for higher protein absorption ability, activation of specific gene expression and intracellular signaling, as well as enhanced cellular interactions. Furthermore, the small pore size of the electrospinning nanofiber network can effectively inhibit the migration of fibroblasts across the barrier, which is vital in GTR/GBR therapies for periodontal regeneration. To obtain dual additives incorporated nanofibers with ideal releasing efficiency and active function, FGM can be fabricated by sequential electrospinning and core-shell structure can be obtained using coaxial electrospinning process.

Appropriate biopolymers and additives should be selected to guarantee their excellent biocompatibility. And biopolymers and additives in proper proportions make it possible to regulate the degradation rate of the membranes. To maintain the membranes in the implanted site for at least 4–6 weeks and avoid collapsing too early, mechanic properties (like flexibility) need to be enhanced. Natural polymers (like chitosan, cellulose, alginate, gelatin, collagen, silk fibroin, zein), with good biological properties and synthetic polymers (like PCL, PLA, PLGA, PBSGL), with good mechanical properties and electrospinnability can be blended to make full use of both advantages.

Capability to promote periodontal regeneration is one of the vital properties required for GTR membranes. Electrospun nanofibers, with inherent ability to mimic natural ECM, perform excellently in inducing osteo-differentiation. Inorganic ceramics like nHA, β-TCP, BGs, ZnO, AuNPs and carbon-based MWNTs are proposed to facilitate the bone regeneration process, and it is possible to enhance mechanical properties at the same time. Furthermore, the functional biomolecules like proteins and growth factors are also utilized to promote regenerative properties, emulating natural *in vivo* osteo-differentiation stimulus. Therefore, aligned electrospun nanofibers can be a promising alternative in organized PDL regeneration.

Infection is regarded as the main factor inducing GTR failure in clinics. Adding multiple drugs facilitates periodontal regeneration and improves the anti-inflammatory microenvironment simultaneously. Till now, various drugs like antibiotics (amoxicillin, ampicillin, metronidazole, tinidazole, doxycycline hydrochloride and tetracycline hydrochloride and combination of amoxicillin-metronidazole-lidocaine, etc.) and NSAIDs, functional proteins like AMPs, oxide components like ZnO and metal nanoparticles like AgNPs, have been incorporated into electrospun nanofibers to inhibit bacterial growing and create ideal anti-inflammatory environment.

Regenerating complex hierarchical structure is vital in periodontal regeneration. Not only alveolar bone should be reconstructed, but also the structure of aligned Sharpey fibers anchoring root cementum to adjacent alveolar bone, which is challenging in hierarchical periodontium regeneration. Although electrospinning technology might be a promising way in tissue regeneration, there are still some problems to be further explored.

Electrospinning technology has distinct advantages in periodontal regeneration. Parameters can be regulated to control relative properties of electrospun fibers, like fiber diameter, porosity and pore size, etc. Various materials including functional polymers and bioceramics, with their respective advantages and disadvantages in physical-chemical characteristics, can be utilized for fabrication. Therefore, it is vital to explore ideal materials in appropriate proportions and optimized parameters for electrospinning process, depending on clinical requirements. Pore size can be controlled by regulating relative parameters during electrospinning process. Relatively big pore size is beneficial for cell infiltration but unfavorable for membrane barrier, while relatively small size leads to opposite characteristic. It is required to strike a balance in pore size, or acquire a multi-layered membrane, one layer with small pore size for membrane barrier and another one with relatively big core size for better cell infiltration.

Electrospun nanofiber membranes usually have a dense inner packing structure, and pore sizes are too small for cells to infiltrate into the mats. Although some methods like salt leaching can improve cell infiltration in electrospun mats, the results are not desirable. Therefore, electrospun mats are widely applied in the GTR field, but not as scaffolds implanted into defected sites. Additionally, vascularization is one of the vital factors in tissue regeneration, because this process supplies essential oxygen and nutrients for cells to proliferate and differentiate. Taken together, the next step is to evaluate the bone regeneration and vascularization *in vivo*.

To maintain the bioactivity and control the releasing profile of drugs polymer-related parameters including component, crystallinity and molecular weight of polymer, and drug-related parameters including molecular weight, drug loading, and crystallinity of drug should be taken into consideration. With the increasingly wide utilization of antibiotics in clinics, bacterial resistance has become a great challenge in bacterial inhibition, thus it is desirable to explore more types of drugs to reduce bacterial resistance, and control periodontal inflammation efficiently. Growth factors degrade quickly *in vivo*, which severely limits their clinical efficiency. Release of the macromolecules based on electrospun nanofibers is not desirable. To construct effective vehicles for controllable release of growth factors, and even realize the temporally distinct release in target period during the regeneration process, electrospinning technology can be combined with other approaches.

Apart from scaffolds, stem cells like PDLCs also play important roles in periodontal tissue engineering. Absence in adequate healthy stem cells is one of the reasons contributing to the incapability of instinctive periodontal regeneration. Stem cells can be cultured on scaffold *in vitro* and then implanted in defected sites to provide sufficient progenitors for tissue regeneration by tissue engineering technology. But the origin of stem cells, the *in vitro* culture condition, the viability of stem cells and clinical effects are challenging for their clinical applications. The next step is to select proper growth factors and stem cells, explore appropriate proportions in scaffolds and improve viability of these stem cells for optimal regeneration of periodontium.

In conclusion, the electrospinning technology has received great attention in periodontal regeneration. Although there still exist some disadvantages and shortcomings to overcome, it is believed that electrospun nanofibers will be further explored and widely applied in clinics for their innate advantages.

## Author Contributions

YZ wrote the manuscript. KL and HY conceived the concept of this review. All authors discussed and commented on the manuscript.

### Conflict of Interest Statement

The authors declare that the research was conducted in the absence of any commercial or financial relationships that could be construed as a potential conflict of interest.
